# Dermoscopic Image Classification of Pigmented Nevus under Deep Learning and the Correlation with Pathological Features

**DOI:** 10.1155/2022/9726181

**Published:** 2022-05-28

**Authors:** Shuang Yang, Chunmei Shu, Haiyou Hu, Guanghui Ma, Min Yang

**Affiliations:** ^1^Department of Dermato-Venereal, Binzhou Medical University Hospital, Binzhou, 256603 Shandong, China; ^2^School of Nursing, Binzhou Medical University, Binzhou, 256603 Shandong, China

## Abstract

The objective of this study was to explore the image classification and case characteristics of pigmented nevus (PN) diagnosed by dermoscopy under deep learning. 268 patients were included as the research objects and they were randomly divided into observation group (*n* = 134) and control group (*n* = 134). Image recognition algorithm was used for feature extraction, segmentation, and classification of dermoscopic images, and the image recognition and classification algorithm were studied as the performance and accuracy of fusion classifier were compared. The results showed that the classifier was optimized, and the linear kernel accuracy was 85.82%. The PN studied mainly included mixed nevus, junctional nevus, intradermal nevus, and acral nevus. The sensitivity under collaborative training was higher than that under feature training and fusion feature training, and the differences among three trainings were significant (*P* < 0.05). The sensitivity of the observation group was 88.65%, and the specificity was 90.26%, while the sensitivity and the specificity of the control group were 85.65% and 84.03%, respectively; there were significant differences between the two groups (*P* < 0.05). In conclusion, dermoscopy under deep learning could be applied as a diagnostic way of PN, which helped improve the accuracy of diagnosis. The dermoscopic manifestations of PN showed a certain corresponding relationship with the type of cases and could provide auxiliary diagnosis in clinical practice. It could be applied clinically.

## 1. Introduction

Pigmented nevus (PN), also known as cellular nevus, is a benign skin tumor that can occur at any age and on any part of the body [1, 2]. PN is mostly black or dark brown, as well as blue-black, black, or normal skin color, light yellow, and dark red; a very small number of PN are colorless [3–5]. Dermoscopy is an emerging technology in the diagnosis and treatment of skin diseases. The accuracy of dermoscopy in diagnosing melanoma is 65-80%. It has been widely applied for pigmented skin diseases, as it can analyze the noninvasive images of the fine structures below the skin surface. It has the advantages of simple operation, noninvasiveness, and easy acceptance by patients [6, 7]. It is difficult to observe the deep skin with the naked eye, but which can be clearly presented with a dermoscope. The dermoscope can project the two-dimensional surface of the tissue structures at different depths, and the pigmentation of the epidermis junction and the superficial dermis as well as the size and shape of blood vessels in superficial vascular plexus can be observed [8, 9]. With the dermoscopy, a corresponding diagnosis for pigmented skin diseases can be given, and a more accurate treatment method for skin diseases can be offered. It expands the scope and depth of the doctor's observation of skin lesions effectively, fills the limitations of visual observation, and provides reliable evidence for clinical diagnosis and treatment [10, 11].

Deep learning can extract low-level features automatically and realize the extraction of advanced features through low-level features [12, 13]. It may retain the information of the image as much as possible for the classification of the images, having a strong generalization ability [14, 15]. On the basis of the learning technology of intelligent machines, image data sets are used for training in the constructed model, and then, predictive analysis is performed on the data not involved [16, 17]. This reflects the powerful data representation of deep learning and also gives a new research method for the image classification [18, 19]. Image classification under deep learning can eliminate useless information in the original image, improve image quality, and greatly improve image classification. In the process of feature extraction, it will also affect the accuracy of the image. A suitable classifier should be used to classify images with feature vectors; thereby, the desired final result can be output [20, 21]. The image fusion algorithm can extract the complementary information of the natural light image and the infrared image, so that a more comprehensive and reliable image describing the same scene can be obtained. Pixel-level fusion refers to the fusion of grayscale images and visible light images, and the image fusion includes the pixel-level-based fusion, feature-based fusion, and decision-based fusion.

With deep learning, the skin lesion area of the dermoscopy image is accurately segmented. The skin lesion area shows different colors, and some colors are close to the skin color. The boundary is diverse with fuzzy shape and irregular appearance. During the imaging, the hair on the skin, natural wrinkles, and bubbles in the dermoscopic image soaking liquid will affect the image processing by the segmentation algorithm. After the feature extraction of the skin lesion area of the segmented image, there are multiple colors presented inside, and the colors are irregular and unevenly distributed. These require more features to fill the defects of feature extraction. Moreover, the intelligent algorithm was used to classify dermoscopic images of PN under deep learning technology, and the correction with pathological features was explored. It provided a reference for the extraction of PN image features and the classification, as well as the diagnosis and treatment of diseases clinically.

## 2. Methods

### 2.1. General Data of Patients

A retrospective analysis was made on the 268 patients, who were diagnosed with PN and underwent dermoscopy on the skin lesions in the hospital from January 2019 to May 2020. The 268 patients were taken as research objects and had histopathological examination. They were randomly divided into observation group (*n* = 134) and control group (*n* = 134). The clinical manifestations, age, gender, and preliminary diagnosis of all patients were complete. The dermoscopic images of patients in the observation group were analyzed under deep learning technology, and those in the control group were processed by conventional method. 213 PNs were observed in the control group and 198 PNs in the observation group. The conventional dermoscopy was used for analyzing images in the control group, while the images were classified by the dermoscopy under deep learning in the observation group. As the general data of patients were compared between the two groups, the difference was not statistically significant (*P* > 0.05) but with a comparability. This study had been approved by the ethics committee of the hospital, and all the included patients signed the informed consent form.

Inclusion criteria are as follows: the patients had skin lesions but no immune system diseases and no infectious diseases. The patients had the ability to speak clearly. They volunteered to participant in. Exclusion criteria are as follows: the patients cannot offer a complete clinical data; the patients went with congenital skin diseases; the patients suffered from diseases of the heart, liver, kidneys, and hematopoietic system, diabetes, or other diseases.

### 2.2. Dermoscopy and Nursing

The digital dermatoscope was used for the examination. The patients should choose a comfortable position, and each patient should make their skin lesions fully exposed. A single lens reflex camera was used to take pictures of the skin lesions under natural light. The lens of dermatoscope was connected with the camera, and the medical ultrasound couplant was applied to the lens of dermatoscope. The surface of the skin lesion was observed with the lens. The lens magnification was 50 times, and the focal length was adjusted. When the image was clear, the image of the electronic dermatoscope was obtained, observed, and saved. The dermatoscopic imaging of patients was evaluated by experienced dermatologists, and two professional doctors made the preliminary diagnostic evaluation.

In the pathological biopsy of skin tissues, disinfection and drape were first performed. When the skin lesion was relatively large, flaps could be designed for suture and banding up. The surgical resection of the skin lesions was performed in the outpatient operating room. Postoperative fixation and dressing change were performed to observe the healing condition of the incision closely. The tissue of the resected skin lesion was fixed with 10% formalin and sliced after a series of steps of dehydration, wax immersion, and embedding. The thickness of the sections was 3 *μ*m. According to the characteristics of skin pathology, experienced skin pathologists performed the classification. PN can be divided into intradermal, mixed, and junctional types. With complete clinical data of patients, comprehensive analysis was performed on dermoscopic characteristics, skin lesion characteristics, onset location, histopathology, and other characteristics.

The psychology of patients should also be cared. If the patients were worried about the pain, the nurses could adopt a gentle and friendly attitude, which would make the patients trust the nurses and let the defense mood go. It was also needed to do a good job in the psychological care of the family members, to eliminate the anxiety and fear of them; and the comfort and encouragement should be given in time. The clinical experience of the surgeon, the success rate of the surgery, and the absence of pain after general anesthesia are needed to be informed to the patients and their family members in details, so that the patients could undergo the surgery in the best condition. Before surgery, the patients were informed with the fasting, water-free, intraoperative position, and precautions for anesthesia cooperation. The nurses prepared all the items needed during the surgery preoperatively, aseptic operation was obeyed strictly during the surgery, and the flow of people in the room was controlled to avoid the incidence of infection. The vital signs of patients were observed at any time. During the surgery, the itinerant nurses cooperated to establish effective venous access, the position was accurately posed, and the light source was adjusted at any time. The massage should be done on the pressured part during the surgery, to prevent the incidence of pressure sores. After the surgery, the attention should be paid on the skin removal and moderate pressure bandaging of the wound in the skin graft area. Saline gauze was used to stop bleeding, electrocoagulation was adopted to stop bleeding for larger bleeding points, and hemostatic gauze was used to stop bleeding in the donation area. The wound was covered and banded with petrolatum gauze. Gentamicin sulfate saline was injected from the needle eye under the flap to wash the wound, and the wound was pressure-wrapped with gentamicin saline gauze pad.

### 2.3. Flow of the Image Recognition Algorithm

Dermoscopic image recognition algorithm included image segmentation, recognition, and feature extraction. The specific algorithm flow was shown in Figure 1. Image edge segmentation included the image preprocessing, the edge segmentation after being denoised, and the removal of hair, bubbles, etc., in the image. After segmentation, the edge was smoothed to obtain the final skin lesion edge.

### 2.4. Recognition and Classification of Dermoscopic Images

In the early years, the recognition and classification of dermatoscopic images mainly depended on human visual judgment. Some special information contained in the image, such as pigment net and blue and white yarn, are used to judge the results. Deep learning is a general term for a type of pattern analysis methods. The neural network system under the convolution operation is just the convolutional neural network. Machine learning is introduced into deep learning, to make it closer to artificial intelligence. Deep learning can obtain more effective information in extracting features. The image classification under deep learning extracted low-level features from the data on its own and then extracted advanced features to realize the accurate classification of images. It saved a lot of manpower and material resources. In recent years, researchers have proposed content-based image classifications to classify images on their visual characteristics such as texture, color, shape, and grayscale.

The activation functions commonly used in network training include Softmax. The activation function can make the network have a strong learning and expressive ability, which is due to the inseparability of some linear issues. When the data was mapped, the interval was 0-1. The Softmax function was shown as

(1) $$\begin{array}{c} \text{f}\left(x\right)=\frac{1}{1+e^{-x}}. \end{array}$$

The derivation equation of Softmax function was expressed as

(2) $$\begin{array}{c} \text{f}\left(x\right)=\left(\frac{1}{1+e^{-x}}\right)=\frac{1}{1+e^{-x}}\left(1‐\frac{1}{1+e^{-x}}\right)=\text{f}\left(x\right)\left(1‐\text{f}\left(x\right)\right). \end{array}$$

It was supposed that the training set *W*(*x*, *y*), *i* = 1, 2 ⋯ , *d* was input, *x* was the *d*-dimensional feature vector, and *y* was the classification label. The samples were divided into two categories, and then, the value of *y* was generally -1 or +1. Equation (3) described the classification of *G*(*x*) training sets.

(3) $$\begin{array}{c} G\left(x\right)=\text{m}•\text{x}+b, \end{array}$$

where *b* was the offset and both *x* and *w* were differential vectors of *d*.

*U* was the classification surface of the farthest hyperplane in the two training sets.

(4) $$\begin{array}{c} G\left(x\right)=\text{m}•\text{x}+b=0. \end{array}$$

The classification surface *U* was obtained by equation (2). If |*G*(*x*)| = 1 was the closest to the classification surface *U*, equation (5) was worked out.

(5) $$\begin{array}{c} {\text{y}}_{i}\left[\left(w•x_{i}+b\right)\right]-1\geq 0,\;\left(\text{i}=1,2,\cdots d\right). \end{array}$$

From equation (3), *U* was proved to be the optimal hyperplane. These vectors that could make the distance closest between the optimal hyperplane and the established sample called support vectors.

With the premise of linear separability, issue solving was performed according to the solution of convex quadratic programming. The Lagrange function was also used with the saddle point, and the Lagrange function was expressed as

(6) $$\begin{array}{c} L\left(\text{w},b,a\right)=\frac{1}{2}{\left\|m\right\|}^{2}-\overset{d}{\underset{i=1}{\sum }}a_{i}\left[y_{i}\left(m•x_{i}+b\right)-1\right]. \end{array}$$

In equation (6), *a* = (*a*1, *a*2, ⋯*ad*)^*T*^ was the Lagrange multiplier vector of sample *x*.

The partial derivative of *m* in the equation was solved. When the partial derivative equaled to zero, equations (7) and (8) were obtained.

(7) $$\begin{array}{c} \frac{\partial L}{\partial b}=0\Rightarrow \overset{d}{\underset{i=1}{\sum }}a_{i}y_{i}=0, \end{array}$$

(8) $$\begin{array}{c} \frac{\partial L}{\partial \text{w}}=0\Rightarrow w=\overset{d}{\underset{i=1}{\sum }}a_{i}y_{i}x_{i}. \end{array}$$

Under invalid constraints, only when the Lagrange multiplier was equal to zero, all valid constraints could be nonzero.

### 2.5. Feature Extraction and Simple Fusion of Dermoscopic Images

Image shape is an important clinical feature. Feature extraction includes area and shape symmetry in the image. Four areas of pixels were used to calculate the center point of the skin lesion area, which was described as

(9) $$\begin{array}{c} {\text{s}}_{\text{pq}}=\overset{\text{rows}}{\underset{i=1}{\sum }}\overset{\text{cols}}{\underset{j=1}{\sum }}i^{p}j^{q}, \end{array}$$

(10) $$\begin{array}{c} \left({\text{r}}_{0},{\text{c}}_{0}\right)=\left(s_{10}/s_{00},s_{01}/s_{00}\right), \end{array}$$

where *S*_pq_ represented the *p* + *q*-th order geometric distance of the image, and the definition of the center distance was expressed as

(11) $$\begin{array}{c} \psi {\text{s}}_{\text{pq}}=\overset{\text{rows}}{\underset{i=1}{\sum }}\overset{\text{cols}}{\underset{j=1}{\sum }}{\left(i‐{\text{r}}_{0}\right)}^{p}{\left(j-c_{0}\right)}^{q}, \end{array}$$

(12) $$\begin{array}{c} L_{1,2}=\left(8\left(\Psi_{02}+\Psi_{20}\pm \left({\left(\Psi_{02}‐\Psi_{20}\right)}^{2}+4\Psi_{11}\right)\frac{1}{2}\right)\right)\frac{1}{2}, \end{array}$$

(13) $$\begin{array}{c} AR=L1/L2. \end{array}$$

The features such as color, texture, and shape contained in the image were fused together to form a new feature set. Both features would produce good classification results when recognizing and classifying. To determine which classification issue should be performed using the kernel function of the SVM classifier, the discriminant functions were expressed as

(14) $$\begin{array}{c} Q\left(\text{x},y\right)=\exp\left\{-{\left|x-y\right|}^{2}/\delta^{2}\right., \end{array}$$

(15) $$\begin{array}{c} \text{f}\left(\text{x}\right)=\mathrm{sgn}\left\{\underset{x_{i}\in sv}{\sum }a_{i}*-Q_{y}\left(\left|x_{i}-x\right|\right)+b*\right\}. \end{array}$$

Equations (9) and (10) were applied to fuse the two feature sets together to form one single feature set. A multiview collaborative training algorithm was proposed, and the characteristics of each feature set were fully utilized.  Figure 2 was from a 48-year-old male patient out of the research objects, with a junctional nevus next to the ear.  Figure 2(a) was the original image before simple image fusion, while Figure 2(b) was the image after processed by the fusion algorithm.

### 2.6. Dermoscopic Image Segmentation

The first step of preprocessing was to segment the image. The method of 0segmentation was just to fuse the results of various segments. Before the algorithm fusion, the image needed to be denoised to avoid noise affecting the image fusion results. After the fusion, the edges of the image were smoothed, which was also a prerequisite for feature extraction. After segmentation, the subdomains of the dermoscopic image were merged, and the obtained image contained the background area and the foreground skin lesion area merely.

After the dermoscopic image was segmented, the *C*_*i*_ color vector of *N* regions was defined as

(16) $$\begin{array}{c} H_{\text{i}}=\left[{\bar{R}}_{i},{\bar{E}}_{i},\bar{B_{i}}\right],\;\left(i=1,2,\cdots ,n\right), \end{array}$$

where ${\bar{R}}_{i}$, ${\bar{E}}_{i}$, and $\bar{B_{i}}$ represented the average of all pixels in si on the three components of the color image, respectively.

*C*_1_ and *C*_2_ represented the two subregions with the largest color distance, so equations (17) and (18) for calculating the image distance were expressed as follows. The images before and after segmentation were shown in Figure 3.

(17) $$\begin{array}{c} L\left(V_{1},V_{2}\right)=\left|V_{1},V_{2}\right|=\sqrt{{\left(\bar{E_{1}}‐\bar{E_{2}}\right)}^{2}+{\left(\bar{G_{1}}‐\bar{G_{2}}\right)}^{2}+{\left(\bar{B_{1}}-\bar{B_{2}}\right)}^{2}}, \end{array}$$

(18) $$\begin{array}{c} \begin{array}{c} \left(C_{1},C_{2}\right)=A\text{rg }\max\left[\text{L}\left({\text{V}}_{C_{1}},{\text{V}}_{C_{2}}\right)\right],\\ C_{1},C_{2}\in \left[1,2,\cdots ,N\right]. \end{array} \end{array}$$

### 2.7. Evaluation Criteria

The true positive (TP) meant that both the results obtained by the instance in the classifier and the actual result were positive. False negative (FN) and false positive (FP) meant that the result obtained by the instance in the classifier was positive, and the actual result was negative. True negative (TN) showed that the result obtained by the instance in the classifier was negative, and the actual result was also negative. The sensitivity stood for the true positive rate, which was expressed as follows:

(19) $$\begin{array}{c} \text{TPR}=\frac{\text{TP}}{\text{TP}+\text{FN}}\times 100\%. \end{array}$$

The specificity stood for the false positive rate, and the expression equation was

(20) $$\begin{array}{c} \text{FPR}=\frac{\text{FP}}{\text{FP}+\text{TN}}\times 100\%. \end{array}$$

### 2.8. Statistical Analysis

Excel and SPASS 21.0 were used to analyze the relevant data of the patients. The measurement data were expressed in the form of $\overset{¯}{x}\pm s$, and the *T* test was also adopted. The enumeration data were expressed as (*n*, %). The distribution of pathological types of different dermoscopic types was analyzed through *χ*^2^ test, with *α* = 0.05 as the test level. When *P* < 0.05, it meant that there was a statistical difference. The statistical method was to analyze the accuracy, sensitivity, and specificity of the dermoscopic diagnosis.

## 3. Results

### 3.1. General Conditions of Patients

There were 268 patients, including 126 males (47.01%) and 142 females (52.99%).  Table 1 showed that the patients with the highest proportion were 18-38 years old, followed by patients 39-58 years old. The proportion of patients aged 6-18 years was the least. There was no significant difference in general data between the two groups (*P* > 0.05).

### 3.2. Result Analysis of the Fusion Algorithm

The classifier was optimized, the input parameter *P* was selected. *P* was the penalty parameter, and the gamma parameter controlled the shape of the kernel, which could control the balance between error minimization and maximization. The accuracy of the three forms of kernel functions was compared, as the result was shown in Figure 4. The accuracy of linear kernel was 85.82%, that of polynomial kernel was 81.96%, and that of the sigmoid kernel was 83.87%. The feature learning of the linear kernel was significantly higher than those of the other two kernels (*P* < 0.05).

The comparison of the AUC of different kernel functions was shown in Figure 5. The AUC of linear kernel was significantly higher than that of polynomial kernel and sigmoid kernel (*P* < 0.05).

### 3.3. Comparison of Training Classification Results

After feature classification, the self-training method was adopted to update the feature classifier. It was shown in Figure 6 that the sensitivity of collaborative training was higher than that of feature training and fusion feature training. There was no significant difference between the results of fusion feature training and collaborative training, but there is no significant difference between feature training and the other two (*P* < 0.05).

### 3.4. Comparison of Sensitivity and Specificity

As shown in Figure 7, the sensitivity and the specificity of the observation group were 88.65% and 90.26%, respectively. The sensitivity of the control group was 85.65%, and the specificity was 84.03%, with significant differences between the two groups (*P* < 0.05).

### 3.5. Skin Lesions

For the 268 patients, there were mainly 4 types of PN, which were mixed, junctional, intradermal, and acral nevi. The distribution of skin lesions was shown in Table 2. Mixed nevus was mainly distributed on the face and the back, junctional nevus was mainly distributed on the face, right ear, and lips, intradermal nevus was mainly on the back and shoulders, and the acral nevus was on the left middle finger and foot.

Figure 8 showed the percentages of cases with the four types. Mixed, junctional, intradermal, and acral nevus accounted for 31.72%, 30.97%, 16.04%, and 21.27%, respectively.

### 3.6. Images of PN Cases with Different Types

The facial image in Figure 9(a) of the mixed nevus was lighter in color, and the shape was irregular. Figures 9(b) and 9(c) were the facial distribution maps of the mixed nevus. The color was black, the shape was round, and the hairs were relatively short.  Figure 9(d) showed that the color of the junctional nevus on lips was light brown. The distribution area was not large, and the shape was irregular. Figures 9(e) and 9(f) had a lighter color, relatively long hairs, and a round shape of junctional nevus on right ear.

Figure 10(a) showed the intradermal nevus with a circular distribution on the back. The color was black and darker in the center, and the edge was brown and lighter. Figures 10(b) and 10(c) displayed the intradermal nevus on shoulders, which were darker in color and were distributed in a circle.  Figure 10(d) was the acral nevus image on foot with lighter color and striped shape, presented as a pattern of parallel grooves. Figures 10(e) and 10(f) displayed the acral nevus on the left middle finger, in dark brown and in stripes.

## 4. Discussion

In clinical application, dermoscopy is simple to operate with low time cost and low expense. It can guide the scope of surgery, which is very helpful in defining the edge of skin lesions. Dermoscopy can also identify many skin lesions of melanoma, and the types of skin lesions can be shown clear under dermoscopy, which is very helpful for the identification of pigmented skin diseases [13, 22]. The key to careful observation of skin diseases is to extract important clues for differential diagnosis. The acra are the high-incidence parts of PN in Asian populations, and the specific shapes can be identified under dermoscopy [23]. The clinical manifestations of PN are relatively diverse. According to histopathological characteristics, PN can be classified into intradermal, mixed, and junctional nevus. Dermoscopy can be taken as an auxiliary diagnostic tool of PN, reducing unnecessary trauma caused by clinical surgical resection effectively. With deep learning technology, the pathological characteristics of patients with PN were classified. The main pathological types of PN in the involved patients included mixed, junctional, intradermal, and acral nevus. Mixed nevi accounted for a highest ratio of 31.72%, and intradermal nevi accounted for 16.04%, which was the least. The distribution of different pathological types of PN was different. Mixed nevi were mainly on the face and back. Junctional ones were mainly on the face, right ear, and lips. Intradermal ones were on the back and shoulders. It was suggested that the algorithm mentioned gave good results for dermoscopic image classification and feature extraction. The skin lesions mainly included the face, back, lips, shoulders, left middle finger, foot, and right ear. In 268 cases, there were more women with PN than men. There were 126 men, accounting for 47.01%, while there were 142 women accounting for 52.99%, which was similar to the results of most studies.

Digital dermoscopy helps dermatologists monitor potential cancerous skin diseases. The effectiveness and accuracy of lesion classification depend on the quality of lesion segmentation. Jamil et al. [24] came up with a new method using wavelet concepts to detect and repair hairs in cancer images. The adaptive sigmoid colon function was used to enhance the contrast between the lesion and the skin. This function focused on the local intensity distribution within a given lesion image. Then, a segmentation method was proposed to segment the lesion accurately from the background. This method was tested on the European Dermoscopy Image Database. The segmentation of skin damage is still a big challenge at current. Because the contrast between the injury and the surrounding skin is low, there are various artifacts and different imaging acquisition conditions. Hwang et al. [25] combined the hybrid model with a new hierarchical structure to segment the melanocyte skin damage in the dermoscopic and standard images. This hybrid method had a segmentation accuracy of 94% on medical skin images, showing certain advantages in the results of standard image segmentation. It also had a high clinical adaptability on the segmentation of melanocyte lesions in dermoscopic images. The image features of the dermoscopy were segmented using the algorithm, and the classifier was optimized. The gamma parameter controlled the shape of the kernel, which can control the balance between error minimization and maximization. The accuracy of linear kernel was 85.82%, and the learning result of linear kernel for feature was significantly higher than those of polynomial kernel and sigmoid kernel (*P* < 0.05). The proposed algorithm showed a good effect on the classification and segmentation of dermoscopic images and also provided a new way for the segmentation of clinical dermoscopic images.

## 5. Conclusion

The intelligent algorithm was used to classify the dermoscopic PN images under deep learning technology, and the correction with pathological features was also explored. The classifier was optimized with a high accuracy. The types of PN were mainly mixed nevus, junctional nevus, intradermal nevus, and acral nevus. The dermoscopic manifestations suggested a certain corresponding relationship with the types of PN, which could provide the auxiliary diagnosis in clinical practice. The algorithm proposed had a certain effectiveness for dermoscopic image segmentation. For the following research, the feature extraction algorithm would be improved, and the confidence of the collaborative algorithm on the result of a single classifier would be studied for image recognition.

## Figures and Tables

**Figure 1:** Flowchart of the image recognition algorithm.

**Figure 2:** Images before and after simple fusion.

**Figure 3:** Dermoscopic images before and after segmentation.

**Figure 4:** Accuracy of feature learning results under different kernel functions. ∗ indicated that the difference was significant as *P* < 0.05.

**Figure 5:** AUC results of feature learning under different kernel functions. ∗ indicated the significant difference with *P* < 0.05.

**Figure 6:** Comparison of training classification results. ∗ indicated that the difference was significant for *P* < 0.05.

**Figure 7:** Comparison of sensitivity and specificity between two groups. ∗ indicated the significant differences, *P* < 0.05.

**Figure 8:** Percentage of cases with four PN types.

**Figure 9:** Images of mixed nevus and junctional nevus.

**Figure 10:** Images of intradermal nevus and acral nevus.

**Table 1:** Comparison of general conditions between the two groups.

Items	Control group	Proportion	Observation group	Proportion	*P*
Age (years old)	46.26 ± 8.51		47.64 ± 5.26		0.766
6-17	19	14.18%	9	6.71%	
18-38	56	41.79%	61	45.52%	
39-58	37	27.61%	38	28.36%	
59-74	22	16.42%	26	19.40%	
Gender					0.494
Male	77	57.46%	49	36.57%	
Female	57	42.54%	85	63.43%	
The total	134		134		

**Table 2:** Types of PN and distribution of skin lesions in patients.

Types	Face	Back	Lips	Shoulders	Left middle finger	Foot	Right ear
Mixed PN	34	51	0	0	0	0	0
Junctional PN	19	0	33	0	0	0	31
Intradermal PN	0	16	0	27	0	0	0
Acral PN	0	0	0	0	32	25	0
The total	53	77	33	27	22	25	31

## Data Availability

The data used to support the findings of this study are available from the corresponding author upon request.
